The article "Application of Different Ventilation Modes Combined with AutoFlow Technology in Thoracic Surgery" was retracted in 2023. Reasons: unreliable results or conclusions; concerns about the data; concerns about the peer review; concerns about the citations.

# Application of Different Ventilation Modes Combined with AutoFlow Technology in Thoracic Surgery

**DOI:** 10.1155/2022/2507149

**Published:** 2022-03-28

**Authors:** Wang Lixian, Yang Yanfang, Cui Chengzong, Jiang Ning, Guo Yufeng

**Affiliations:** Cangzhou Central Hospital, Cangzhou, China

## Abstract

To investigate the effect of AutoFlow on airway pressure and hemodynamics in mechanical ventilation constant volume-control ventilation mode, 100 patients receiving mechanical ventilation were randomly divided into observation group (SIMV-PSV-PEEP + AutoFlow) and control group (SIMV-PSV-PEEP). The results showed that the peak airway pressure and average airway pressure decreased with different flow rate settings and automatic flow conversion (*P* < 0.05). The peak airway pressure and mean airway pressure decreased with different resistance settings (*P* < 0.05). With different compliance settings, the peak airway pressure and average airway pressure decreased after being assisted with an automatic converter (*P* < 0.05). Adding AutoFlow on the basis of SIMV-PSV mode can significantly reduce peak inspiratory pressure (PIP), mean airway pressure (P_mean_), and airway resistance (R). There was no significant difference in hemodynamic monitoring results between the observation group and the control group. It is proved that the SIMV constant volume-controlled ventilation mode combined with AutoFlow can not only ensure tidal volume but also avoid excessive airway pressure, which has little effect on hemodynamics.

## 1. Introduction

At present, ventilator technology tends to mature and the application level of clinicians is stable. Mechanical ventilation has been widely used and has become an important means of clinical treatment and rescue of critically ill patients. With the accumulation of clinical experience and the application of microcomputer technology, some new mechanical ventilation modes and technologies have been developed and applied, such as: its common features are that compared with the previous auxiliary ventilation mode, it is closer to the physiological state, more in line with the actual respiratory mechanical characteristics and pathophysiology of patients, and more humanized. Under the condition of meeting the ventilation, it aims to make patients comfortable to the greatest extent, pay more attention to preserving patients' autonomous breathing function, improve man-machine coordination as much as possible, minimize patients' respiratory work, and avoid complications related to artificial respiration support [1, 2]. Traditional fixed pressure ventilation mode BiPAP is applied to neonates. Because of constant pressure, improper pressure adjustment, or increased airway resistance, it is easy to lead to insufficient ventilation, causing hypoxemia and carbon dioxide retention. The auxiliary ventilation technology combined with SIMV + AutoFlow can dynamically adjust the air flow according to the patient's current airway pressure and chest-lung compliance and send the preset tidal volume with a deceleration wave and the lowest pressure, which can make up for the deficiency of the BiPAP mode [3].

The article "Application of Different Ventilation Modes Combined with AutoFlow Technology in Thoracic Surgery" was retracted in 2023. Reasons: unreliable results or conclusions; concerns about the data; concerns about the peer review; concerns about the citations.

## 2. Literature Review

Ge et al. believed that thoracoscopy is a new technology applied in thoracic surgery in recent years. Under the direct vision of a high-definition television imaging system, the operation system is inserted into the chest through chest wall incision to diagnose and treat chest diseases. This operation has the advantages of small incision, small injury, and fast recovery and can be widely used in clinics [4]. Campos and Sharma believed that patients with primary bronchial lung cancer (referred to as lung cancer) and chronic obstructive pulmonary disease (COPD) had common risk factors, such as smoking, so many lung cancer patients were diagnosed with COPD in the preoperative pulmonary function assessment of thoracoscopy [3]. Hahm believe that patients often have complications such as pulmonary infection and atelectasis after thoracoscopic surgery due to low ciliary function, which increases the length of hospital stay, so it puts forward higher requirements for nursing work [5]. Gedik and Alar believed that each pressurization of the oscillating sputum drainage system can force the air flow to quickly pass through the lung tissue, stimulate the cilia through the chest wall oscillation, improve the cilia swing frequency, promote the secretion to fall off from the trachea and bronchus and move to the oral cavity, and discharge it through normal cough or negative pressure sputum suction after reaching the oral cavity [6]. Meng et al. believed that this method is suitable for patients with pulmonary insufficiency caused by difficulty in excreting pulmonary secretions or mucus blocking the lungs and can promote airway clearance and sputum excretion or improve bronchial drainage. Therefore, it can reduce the incidence of pulmonary infection and atelectasis in patients with lung cancer complicated with COPD [7]. Habertheuer et al. thought that volume-controlled ventilation (VCV) and pressure-controlled ventilation (PCV) are commonly used in mechanical ventilation (MV). VCV and PCV have their own advantages and disadvantages. The main advantage of VCV is to ensure tidal volume, while PCV has obvious advantages in reducing the risk of barotrauma, improving human-machine coordination, reducing patients' respiratory work, and improving gas distribution in the lung and ventilation blood flow ratio [8]. Park believes that the automatic flow function of the ventilator is a kind of dual control mode. The dual control mode attempts to combine the advantages of VCV and PCV. Some studies have compared the differences between other dual control modes and traditional constant current air supply VCV and PCV. It is considered that the advantages of a dual control mode are as follows: while ensuring the tidal volume, it avoids the disharmony between the air supply flow rate caused by the fixed VCV flow rate and the needs of patients, improves the man-machine synchronization, reduces the patient's respiratory work, reduces airway pressure, improves gas exchange, and is safer for patients with unstable ventilation. However, few studies comprehensively compare the changes of airway pressure, flow rate, and other respiratory mechanical indexes after auxiliary automatic conversion [1]. George et al. believed that the study of a model lung can set different compliance, resistance, and inspiratory flow rate and exclude the influence of patients' breathing mode and other clinical conditions. It has good repeatability and is an ideal method to study respiratory mechanics [9]. Rohde et al. believed that AutoFlow is an auxiliary ventilation technology combined with the SIMV mode. It is not an independent ventilation mode, but a functional extension of the capacity control breathing mode [10]. Dearani et al. believed that after using AutoFlow, the ventilator will dynamically adjust the air flow according to the patient's current airway pressure and chest lung compliance and send it to the preset tidal site with the velocity waveform of deceleration wave and the lowest pressure, so as to avoid the occurrence of barotrauma to the greatest extent. At the same time, the patient is allowed to breathe freely in the whole ventilation cycle, and the man-machine coordination is better. If the airway resistance and chest-lung compliance change, the airway pressure shall be increased or decreased by 3 cm H_2_O each time, but not higher than 5 cm H_2_O below the set pressure alarm high limit, otherwise the pressure and tidal volume alarm [11].

The article "Application of Different Ventilation Modes Combined with AutoFlow Technology in Thoracic Surgery" was retracted in 2023. Reasons: unreliable results or conclusions; concerns about the data; concerns about the peer review; concerns about the citations.

Based on the current research, in order to explore the effect of AutoFlow on airway pressure and hemodynamics in mechanical ventilation constant volume control ventilation mode, 100 patients receiving mechanical ventilation were randomly divided into observation group (SIMV-PSV-PEEP + AutoFlow) and control group (SIMV-PSV-PEEP).

## 3. Materials and Methods

### 3.1. Clinical Data

From January 2019 to January 2021, 100 patients with respiratory failure received mechanical ventilation in the respiratory intensive care unit (RICU) of our hospital, including 75 males and 25 females. All patients underwent oral endotracheal intubation or tracheotomy after admission to the RICU and were mechanically ventilated with the Drager EVTA 4 ventilator. The ventilation mode was SIMV pressure support ventilation (PSV)-positive end expiratory pressure (PEEP) [12].

### 3.2. Method

#### 3.2.1. When Transferred to ICU

In a randomized controlled study, the included children were randomly divided into groups A and B according to the random number table. Group A represents the BiPAP group and group B represents the SIMV + AutoFlow group. After general anesthesia, the subjects of the two groups were transferred to the ICU under stable respiratory and circulatory conditions, such as body temperature, heart rate, blood pressure, oxygen saturation, central venous pressure (CVP), respiratory rate, tidal volume, and peak airway pressure and resistance, and mechanical ventilation was given with the German Drager EVTA 4 ventilator.

#### 3.2.2. Breathing Mode Using Ventilator

BiPAP ventilation mode parameter setting: determine the tidal volume (VT) by adjusting the difference between P_high_ and P_low_ according to the patient's weight, which is generally calculated as TV = 8 ∼ 10 ml/kg. The preset respiratory rate is 25 ∼ 40 times/min. Adjust the inspiratory time to determine the inspiratory respiratory ratio (I:e), usually 1 : 1 or 1 : 2; P_high_ is usually 15 ∼ 20 cm H_2_O, plot is 5 ∼ 7 cm H_2_O. SIMV + AutoFlow ventilation mode parameter setting: the respiratory rate is usually 25 ∼ 40 times/min, VT = 8 ∼ 10 ml/kg, the tidal volume is set, the breathing ratio is set from 1 : 1 to 1 : 2, and the positive end expiratory pressure (PEEP) is generally set at 0 ∼ 3 cm H_2_O. The support pressure (PSV or P_ASB_) is generally adjusted to 10 ∼ 20 cm H_2_O. After the ventilator is connected with the patient, the ventilation parameters are adjusted appropriately according to the specific condition [13].

#### 3.2.3. Offline Standard

When the patient is awake and cooperative, spontaneous breathing is stable, cough and swallowing reflexes are recovered, the respiratory tract is unobstructed, circulation is stable, and the internal environment is balanced. It is expected that there is no possibility of reoperation and endotracheal intubation, and the offline steps can be implemented when the blood gas analysis Pao is > 60 mmHg, PaCO_2_ is < 50 mm Hg, and FiO_2_ is ≤ 40%.

#### 3.2.4. Offline Steps

Firstly, reduce the inhaled oxygen concentration to less than 40%, and then, gradually adjust the support pressure to less than 5cmho. The respiratory rate in the SIMV mode is gradually reduced to less than 5 times per minute, the P_high_ in the BIPAP mode is gradually reduced, the P_low_ is synchronously reduced, and the reduction can be stopped when it reaches 3 cm H_2_O. When the difference between P_high_ and P_low_ is reduced to 5 ∼ 7 cm H_2_O, it can be changed to CPAP or maintained at 5 cm H_2_O and the P_ASB_ can be synchronously reduced to less than 5 cm H_2_O. Observe for 30 minutes after the trial shutdown and measure the arterial blood gas analysis (including arterial blood gas pH value, arterial blood oxygen partial pressure, arterial blood carbon dioxide partial pressure, blood oxygen saturation, and BE value). The patient's blood pressure, heart rate, and respiration are stable. Endotracheal intubation was pulled out, and oxygen was absorbed by a mask. After tracheotomy, patients were removed from the machine, oxygen was directly absorbed by gas cut masks to ensure normal blood oxygen saturation [14].

The article "Application of Different Ventilation Modes Combined with AutoFlow Technology in Thoracic Surgery" was retracted in 2023. Reasons: unreliable results or conclusions; concerns about the data; concerns about the peer review; concerns about the citations.

### 3.3. Observation Indicators

Monitoring indicators include the following: (1) record the general information of patients after admission to the ICU, including patient name, gender, age, weight, hospitalization number, admission diagnosis, operation status, operation name, and cardiopulmonary bypass time and (2) after admission to the ICU, each patient was continuously monitored for basic vital signs, including body temperature, blood pressure, heart rate, pulse, respiratory rate, and blood oxygen saturation. After admission, routine arterial blood gas analysis was given. Vital signs, blood gas (pH, PaCO_2_, and PaO_2_), and ventilator indexes, including respiratory rate (f), tidal volume (VT), peak airway pressure (P_peak_), lung compliance (c), airway resistance (*R*), and minute ventilation (MV), were recorded at five time points of admission (t0), 30 minutes (t1), one hour (t2), two hours (t3), and three hours (t4).

### 3.4. Statistical Treatment

All data were processed by PEMs 3.1 medical statistics software package, the observation data were expressed by *X* ± *s*, and the paired *t*-test was used for comparison between groups. *P* < 0.05 was statistically significant.

## 4. Results

The respiratory mechanics results of the two groups are shown in Table 1. Table 1 shows that PIP and P_mean_ in the observation group decreased significantly and *R* decreased significantly compared with the control group. There was no significant difference in VT between the observation group and the control group. The results of hemodynamics and arterial blood gas analysis of the two groups are shown in Tables 2 and 3. It can be seen from Tables 2 and 3 that there is no significant difference in arterial blood gas analysis results and hemodynamic monitoring results between the two groups [15].

The article "Application of Different Ventilation Modes Combined with AutoFlow Technology in Thoracic Surgery" was retracted in 2023. Reasons: unreliable results or conclusions; concerns about the data; concerns about the peer review; concerns about the citations.

A total of 100 children were enrolled. The longest transfer time was 137 minutes, and the longest use time of ventilator was 40 hours and the shortest was 5 hours. Five cases died recently after operation, including 3 cases of low cardiac output syndrome, 1 case of arrhythmia, and 1 case of pulmonary infection.

Two independent samples *t*-test was used for the general data of the two groups. Among the 100 patients observed, there was no significant difference in age, weight, transit time, blocking time, vital signs, and ventilator monitoring indexes between the two groups (*P* > 0.05).

The intragroup comparison showed that there was significant difference in peak airway pressure at different time points in patients with the same mechanical ventilation mode with time (*P* < 0.05). It can be seen from the figure that the peak airway pressure of children applying the SIMV + AutoFlow mechanical ventilation mode is lower than that of the BiPAP group and shows a downward trend (see Figure 1 for the results) [16]. At the same time, the alveolar compliance was different at different time points (*P* > 0.05) (see Figure 2 for the results).

The delivered tidal volume remained unchanged before and after auxiliary automatic conversion (500 ± 1.3 ml vs, 500 ± 1.2 ml, *P* > 0.05). After auxiliary automatic conversion, peak airway pressure and average airway pressure decreased (*P* < 0.05) (see Figure 3).

On the premise that the conveying moisture volume remains unchanged (*P* > 0.05), with different flow rate settings, the peak airway pressure and average airway pressure decreased after auxiliary automatic flow conversion (*P* < 0.05) (see Figures 4 and 5); with different resistance settings, the peak airway pressure and average airway pressure decreased after auxiliary automatic flow conversion (*P* < 0.05) (see Figures 6 and 7); with different compliance settings, the peak airway pressure and average airway pressure decreased after assisted automatic flow conversion (*P* < 0.05) (see Figures 8 and 9).

## 5. Discussion

Mechanical ventilation modes can be divided into two categories: constant pressure ventilation and constant volume ventilation (SIMV). Compared with constant pressure ventilation, the advantage of constant volume ventilation is that it can ensure the preset tidal volume; the doctor presets the VT delivered by the command breathing mode, and then, the ventilator delivers the predetermined VT regardless of resistance and compliance. The proximal airway pressure of patients changes. If the airway resistance increases or the respiratory compliance decreases, it can cause high peak airway pressure and plateau pressure, resulting in excessive expansion of localized alveoli and barotrauma [17]. The data of this group showed that after SIMV combined with AutoFlow, the peak inspiratory pressure and average airway pressure decreased significantly and the airway resistance decreased, indicating that AutoFlow can improve respiratory mechanics to a certain extent. AutoFlow itself is not an independent ventilation mode. As a pressure regulation function extension of the volume-controlled breathing mode, it combines the advantages of pressure-controlled ventilation and volume-controlled ventilation when used in combination with the SIMV mode. The working principle is as follows: at the beginning of the ventilator, four consecutive experimental breaths with a pressure of 10 cm H_2_O are performed, and the current airway pressure and lung-chest compliance of the patient are continuously measured by a microcomputer. According to the volume-pressure relationship, calculate the suction pressure required for the next ventilation to reach the preset tidal volume, automatically adjust the preset suction pressure level (usually adjusted to 75% of the calculated value), and send the preset tidal volume with the velocity waveform of deceleration wave and the lowest pressure so as to make the actual tidal volume consistent with the preset tidal volume and avoid the occurrence of air pressure injury to the greatest extent [18, 19]. At the same time, the patient is allowed to breathe freely throughout the ventilation cycle. The inspiratory pressure level can be automatically adjusted within the range of 5 cm H_2_O when the end expiratory airway pressure reaches the preset inspiratory upper limit pressure level, but each adjustment range is less than 3 cm H_2_O, otherwise the pressure and tidal volume alarm. The main advantages of SIMV combined with AutoFlow are as follows: good man-machine coordination can reduce or avoid the use of sedatives or muscle relaxants; it can automatically adjust the inspiratory pressure according to the monitoring indicators of lung function and meet the preset tidal volume with the lowest airway pressure, which is conducive to the prevention of barotrauma. The waveform of air flow velocity is a deceleration wave. When the airway is blocked, it can reduce eddy current, so as to reduce pressure consumption and reduce inspiratory peak pressure [20, 21].

The article "Application of Different Ventilation Modes Combined with AutoFlow Technology in Thoracic Surgery" was retracted in 2023. Reasons: unreliable results or conclusions; concerns about the data; concerns about the peer review; concerns about the citations.

AutoFlow is suitable for some patients with respiratory failure (such as acute respiratory distress) and high airway resistance (such as critical asthma). According to the actual situation of the patient, on the premise of avoiding air pressure injury, the preset inspiratory upper limit pressure level should not be too low; otherwise, it can be difficult to reach the preset tidal volume because the range of inspiratory pressure automatically adjusted by the computer is too small [22]. The data of this group show that there is no significant difference in hemodynamic monitoring parameters between the observation group and the control group after being combined with AutoFlow, indicating that SIMVP combined with AutoFlow has little effect on hemodynamics [23–25].

## 6. Conclusion

Compared with BiPAP, the SMV + AutoFlow mechanical ventilation mode can significantly reduce peak airway pressure and increase lung compliance. Peak airway pressure decreases and lung compliance increases with time. Using the BIPAP mode and the SIMV + AutoFlow breathing mode, there was no significant difference in arterial blood gas, tidal volume, minute ventilation, and airway resistance. SIMV + AutoFlow is a safe and reliable mechanical ventilation mode for patients with congenital heart disease and deformity after correction.

## Figures and Tables

**Figure 1:** Change in the trend of peak airway pressure in the SIMV + AutoFlow group at different time points.

**Figure 2:** Change in the trend of lung compliance in the SIMV + AutoFlow group at different time points.

**Figure 3:** Peak and average airway pressure before and after auxiliary automatic conversion.

**Figure 4:** Changes in peak airway pressure after auxiliary automatic conversion under different flow rate settings.

**Figure 5:** Changes in mean airway pressure after auxiliary automatic conversion under different flow rate settings.

**Figure 6:** Changes in peak airway pressure before and after auxiliary automatic conversion under different resistance settings.

**Figure 7:** Changes in mean airway pressure before and after auxiliary automatic conversion under different resistance settings.

**Figure 8:** Changes in peak airway pressure before and after auxiliary automatic conversion under nonreturn compliance modification.

**Figure 9:** Changes of mean airway pressure before and after Fuchuan automatic conversion under different compliance settings.

**Table 1:** Respiratory mechanics results of two groups (*x* ± *s*).

Group	Number of cases	PIP	P_mean_	R	VT
Observation group	50	28 ± 5	27 ± 4	40 ± 18	589 ± 70.1
Control group	50	15 ± 4	9 ± 4	26 ± 14	574 ± 79.9
*P* value		<0.01	<0.05	<0.05	>0.05

**Table 2:** Blood gas and hemodynamic results of two groups.

Group	Number of cases	HR	ABPM	PH	PaO_2_
Observation group	50	95 ± 11	74 ± 12	6.9 ± 0.1	87 ± 13
Control group	50	92 ± 10	72 ± 10	6.9 ± 0.1	91 ± 16
*P* value		>0.05	>0.05	>0.05	>0.05

The article "Application of Different Ventilation Modes Combined with AutoFlow Technology in Thoracic Surgery" was retracted in 2023. Reasons: unreliable results or conclusions; concerns about the data; concerns about the peer review; concerns about the citations.

**Table 3:** Blood gas and hemodynamic results of the two groups.

Group	Number of cases	PaCO_2_	CVP	CO	SV
Observation group	50	43 ± 10	14.8 ± 3.1	7.6 ± 0.9	65 ± 10.4
Control group	50	41 ± 9	15.4 ± 3.0	7.8 ± 0.8	65 ± 8.9
*P* value		>0.05	>0.05	>0.05	>0.05

## Data Availability

The data used to support the findings of this paper are available from the corresponding author upon request.
